# Development of an *in Vitro* System to Simulate the Adsorption of Self-Emulsifying Tea (*Camellia oleifera*) Seed Oil 

**DOI:** 10.3390/molecules21050479

**Published:** 2016-04-29

**Authors:** Issara Sramala, Wichchunee Pinket, Pawinee Pongwan, Suwatchai Jarussophon, Kittiwut Kasemwong

**Affiliations:** Nano Agro and Food Innovation Laboratory, National Nanotechnology Center (NANOTEC), National Science and Technology Development Agency (NSTDA), 111 Thailand Science Park, Phahonyothin Road, Khlong Nueng, Khlong Luang, Pathumthani 12120, Thailand; wichchunee@nanotec.or.th (W.P.); pawinee@nanotec.or.th (P.P.); suwatchai@nanotec.or.th (S.J.); kittiwut@nanotec.or.th (K.K.)

**Keywords:** self-emulsifying oil formulations, *Camellia oleifera*, lecithin, surfactant blends, oil adsorption

## Abstract

In this study, tea (*Camellia oleifera*) seed oil was formulated into self-emulsifying oil formulations (SEOF) to enhance the aqueous dispersibility and intestinal retention to achieve higher bioavailability. Self-emulsifying tea seed oils were developed by using different concentrations of lecithin in combination with surfactant blends (Span^®^80 and Tween^®^80). The lecithin/surfactant systems were able to provide clear and stable liquid formulations. The SEOF were investigated for physicochemical properties including appearance, emulsion droplets size, PDI and zeta potential. The chemical compositions of tea seed oil and SEOF were compared using GC-MS techniques. In addition, the oil adsorption measurement on artificial membranes was performed using a Franz cell apparatus and colorimetric analysis. The microscopic structure of membranes was observed with scanning electron microscopy (SEM). After aqueous dilution with fed-state simulated gastric fluid (FeSSGF), the droplet size of all SEOF was close to 200 nm with low PDI values and the zeta potential was negative. GC-MS chromatograms revealed that the chemical compositions of SEOF were not significantly different from that of the original tea seed oil. The morphological study showed that only the SEOF could form film layers. The oil droplets were extracted both from membrane treated with tea seed oil and the SEOF in order to evaluate the chemical compositions by GC-MS.

## 1. Introduction

Self-emulsifying delivery systems (SEDS) are vital tools used to improve the solubility and bioavailability of lipophilic bioactive compounds. These systems can form fine oil-in-water (o/w) emulsions when introduced into an aqueous phase, such as gastrointestinal fluids, under mild agitation [1,2]. For oral administration, self-emulsifying oil formulations (SEOF) are designed to be safe for consumption by using only food compatible ingredients. Lecithin is a good choice for the development of SEOF because of its GRAS status, biodegradability and low cost. It is also desirable for use as a good surface active agent in food applications. However, the use of lecithin tends to form liquid crystal phases that promote the formation of undesirable emulsions [3]. This limitation has been overcome with the introduction of surfactants or blends of surfactants that show a synergistic effect with lecithin in microemulsion systems.

Tea (*Camellia oleifera*) seed oil, one of the most important edible oils, is an excellent source of unsaturated fatty acids. It has been reported that tea seed oil provides great health benefits due to its high oleic acid composition [4,5]. It also contains a variety of bioactive components, such as vitamin E, phytosterols, squalene and flavonoids. Several studies have reported that the consumption of tea seed oil provides significant health-promoting effects. Long-term intake is helpful in preventing coronary heart disease, cancer, arteriosclerosis, and increasing gastrointestinal absorption function [4,6].

In this work, the SEOF of tea (*Camellia oleifera*) seed oils were developed with aim of increasing its dispersibility and intestinal retention to achieve higher bioavailability. Figure 1 shows a proposed mechanism where self-emulsified oil droplet could be adsorbed onto an unstirred mucus glycogalyx layer and epithelial brush border of the gut lumen. The localized oil droplet would not move along with dietary content in gut lumen. As the intestinal retention of the nutrient was increased, the bioavailability could also be increased [7,8,9,10].

The self-emulsifying tea seed oil was formulated with soy lecithin in combination with surfactant blends (Span^®^80 and Tween^®^80). The appearance, emulsion droplets size, PDI and zeta potential of developed formulations were studied. A GC-MS analysis was performed to investigate the chemical compositions of SEOF in comparison with the original tea seed oil. In addition, the SEOF was also evaluated for oil adsorption on artificial membranes by using a Franz cell apparatus and scanning electron microscopy (SEM).

## 2. Results

### 2.1. Ternary Phase Diagram

The ternary phase diagram for the systems prepared with tea seed oil containing different concentrations of lecithin and surfactant blends (Span^®^80/Tween^®^80 ratio of 1:1) is shown in Figure 2. The grey region represents yellowish clear tea seed oil liquids when formulated into SEOF. It was observed that the combination of hydrophilic and lipophilic surfactants alone could not provide isotropic liquids when mixed with tea seed oil. On the other hand, the use of an appropriate concentration of lecithin in combination with surfactant blends could provide yellowish clear liquids.

### 2.2. Droplet Size and Zeta Potential Determination

To compare dispersibility of the prepared formulations at their equilibrium state, a series of SEOF were prepared based on the isotropic region in the ternary phase diagrams. High loading of tea seed oil concentration was required in order to achieve its nutritional and pharmaceutical values for the SEOF. All formulas are highlighted in Figure 2b, consisting of formulations A1–A3 (yellow marks), B1–B3 (blue marks), C1–C3 (red marks) and D1–D3 (green marks). Each formulation was vigorously mixed until its equilibrium state was reached. After aqueous dilution with fed-state simulated gastric fluid (FeSSGF) at pH 6.4, the droplet sizes of all formulations were close to 200 nm with low PDI values (<0.3). As shown in Table 1, the zeta potential was found to be negative in a range between −6.16 to −20.39 mV. The higher loading concentration of surfactant blends (nonionic surfactant) in the formulations causes an increase of their zeta potential close to 0 mV. Based on these results, we select A1 as the optimal formula because their droplets size and PDI value were not significantly different when compared to the formulations with higher lecithin and surfactant blends concentration. The selected formula was further used for chemical composition analysis and oil adsorption measurements. The appearance of SEOF (A1) compared with tea seed oil is shown in Figure 3.

### 2.3. Fatty Acid Composition

To evaluate the stability of fatty acids (major component) presented in self-emulsifying tea seed oil formulation, the GC-MS chromatograms of tea seed oil and SEOF (A1) were recorded as shown in Figure 4. It was found that the fatty acid composition profile of SEOF was not significantly different from that of the original tea seed oil. The results also showed a variety of fatty acids, consisting of palmitic acid (C16:0), stearic acid (C18:0), oleic acid (C18:1) and linoleic acid (C18:2).

Remarkably, the highest levels of unsaturated oleic acid (80.64%–82.17%) were found in both of tea seed oil and SEOF, followed by palmitic acid (8.83%–9.01%), linoleic acid (7.64%–8.83%), and stearic acid (1.37%–1.52%) as shown in Table 2.

The quantity and the GC-MS profile of fatty acids were monitored, and the profile did not change over time for three months, as shown in Table 3. In fact, clear solution of SEOF was still observed while there was some solid precipitate in the original tea seed oil.

### 2.4. In Vitro Study of Oil Adsorption

Figure 5 showed the appearance of membrane after performed in a Franz cell apparatus. It was found that the red color of Oil Red O (oil-soluble dye) was located on the membrane surface with SEOF. Moreover, the intensity of red color increased as the operating time increased. In case of tea seed oil (used as a positive control), there was no difference between the appearance of fresh membrane and membrane after the oil adsorption study over a 24 h period.

The surface and structure morphology of the cellulose acetate membrane were investigated by scanning electron microscopy. As can be seen in Figure 6c, there is a large amount of oil film layers adsorbed in the pores of membrane performed with SEOF. On the other hand, oil film layer was not observed on membrane surface treated with tea seed oil as shown in Figure 6b. Also, its pore structure was clearly visible similar to a blank membrane without any treatment (Figure 6a).

The oil droplets were extracted both from membrane treated with tea seed oil and the SEOF in order to evaluate the chemical compositions by GC-MS. It was found that only the membrane treated with SEOF showed the existence of fatty acids remaining on the membrane surface (Figure 7). This observation suggested that the absorption of fatty acids of the stable SEOF tends to be enhanced by surface membrane retention.

## 3. Discussion

In this work, lecithin-surfactant systems were formulated to produce self-emulsifying tea seed oils. Ternary phase diagrams were constructed to identify the range of the isotropic region and optimize the concentration of tea seed oil, lecithin and surfactant blends for the development of SEOF. It was found that only suitable concentrations of tea seed oil, lecithin and surfactant blends will be able to produce a stable SEOF. This could be explained on the basis that Tween^®^80 which is a hydrophilic surfactant (HLB = 15) can induce an immiscible oil/surfactant [11]. When we added the lecithin into the system, the unsaturated tails of lecithin and Tween^®^80 help them to interact synergistically with each other leading to a tight packing at the surface of the oil [12]. Furthermore, it has been found that lecithin-based microemulsion formulation with co-surfactant provided an excellent oil solubilization capacity for a wide range of oils [13,14]. Recent formulation developments rely on free energy rather than HLB values [15,16,17]. Droplet size measurements indicated that the lecithin-surfactant systems can produce nanosized droplets with narrow size distribution, leading to an increase of the emulsion stability. The charge on an oil droplet is negative due to the presence of free fatty acids in the formulation [1,18].

The fatty acid composition of tea seed oil is representative of its quality and potentiality. It has been found in this study that tea seed oil contained both saturated (palmitic acid and stearic acid) and unsaturated fatty acids (oleic acid and linoleic acid). High levels of oleic acid were observed in this oil. Su *et al.* reported that the major fatty acid found in tea (*Camellia* species) seed oil was oleic acid, with levels ranging between 41.1% and 89.0%, depending on sample collection locations. The presence of high amounts of oleic acid gives tea seed oil better health-promoting effects and higher storage stability [5].

The main purpose of SEDS was to improve the poor aqueous solubility of active compounds because this property is considered one of the prerequisites for intestinal absorption [19]. These systems easily form fine emulsions when subjected to the gastrointestinal tract environment. In our work, the *in vitro* study of oil adsorption on artificial membranes were carried out for the optimal SEOF compared with original tea seed oil (control). When tea seed oil was formulated into SEOF, it was found that oil droplets remained suspended in the simulated GI fluid until the end of the run and some oil droplets were adsorbed on the membrane surface. It could be suggested that the SEOF has the potential to enhance the aqueous dispersibility and increase the contact area between oil droplets and membrane surface.

## 4. Materials and Methods

### 4.1. Chemicals

The tea seed oil was obtained from the Tea Oil and Plant Oils Development Center, Chaipattana Foundation (Chiang Rai, Thailand). Soy lecithin fluid was obtained from Rama Production Co., Ltd. (Bangkok, Thailand). Tween^®^80, Span^®^80, Oil Red O and sodium phosphate tribasic dodecahydrate were purchased from Sigma-Aldrich Co. (St. Louis, MO, USA). Hydrochloric acid (37%), sodium chloride and sodium hydroxide were purchased from CARLO ERBA Reagents S.A.S. (Val de Reuil, France). Deionized water was used for the preparation of all the solutions.

### 4.2. Construction of Ternary Phase Diagram

Ternary phase diagrams were constructed according to the preparation of various formulations containing different ratios of tea seed oil, lecithin and surfactants blends (Span^®^80/Tween^®^80 ratio of 1:1). In our case, we used a hydrophilic surfactant (Tween^®^80) to exhibit polar characteristics in the system. Each formulation was stirred thoroughly for 5 h (500 rpm) and kept at ambient temperature overnight. Finally, the prepared formulations were observed for their appearance and categorized as isotropic mixtures in the phase diagram when they were yellowish clear liquids.

### 4.3. Preparation of Self-Emulsifying Oil Formulations (SEOF)

Series of formulations comprising different concentrations of tea seed oil, lecithin and surfactant blends (Span^®^80/Tween^®^80 ratio of 1:1) were prepared based on the ternary phase diagram. The mixtures were added in clear glass vials and thoroughly stirred at 500 rpm overnight.

### 4.4. Emulsion Droplet Size and Zeta Potential Measurement

The SEOF were diluted 1000-fold with fed-state simulated gastric fluid (FeSSGF) pH 6.4 as described by Jantratid *et al*. [20], mixed by a vortex mixer and analyzed using a Zetasizer (Zetasizer Nano ZS, Malvern, Worcestershire, UK) in order to evaluate emulsion droplet size, PDI and zeta potential. All study experiments were conducted in triplicate to ensure reproducibility and the mean values were reported.

### 4.5. Chemical Composition Analysis

The tea seed oil and SEOF were methylated to methyl ester by HCl-methanol and extracted by toluene. The fatty acids were analyzed by Gas Chromatography-Mass Spectrometry (GCMS-QP2010 Ultra, Shimadzu Co., Kyoto, Japan) equipped with DB-wax column, with dimensions of 30 m × 0.32 mm × 0.25 μm film thickness (Agilent Technologies, Santa Clara, CA, USA). Fatty acid composition was expressed as a percentage of total fatty acids.

### 4.6. InVitro Study of Oil Adsorption

A Franz cell apparatus was used to determine the oil adsorption on artificial membranes according to the method of Cascone *et al.* [21] with some modification. A buffer solution (pH 6.8) was filled in the receptor compartment and covered with cellulose acetate membrane (pore size 0.2 μm) followed by a silicone o-ring on the top. The matched donor compartment was mounted and filled with sample solutions, prepared by adding Oil Red O (0.5 mg) into tea seed oil or SEOF (20 μL) in order to visualize the oil adsorption on membrane surface. The resulting solutions were then diluted with buffer solution at pH 6.8 (3 mL) before performing the Franz cell experiments. All openings of donor and receptor compartment were enclosed with aluminum foil and Parafilm. The experiments were performed at 37 °C with continuous stirring. Membranes were withdrawn at predetermined time intervals and rinsed with deionized water. To evaluate the adsorption of oil, the morphology of membrane surface was observed under scanning electron microscope (Hitachi S-3400N, Hitachi High-Technologies Co., Tokyo, Japan) and the chemical composition of adsorbed oil on the membrane was determined by the GC-MS technique.

### 4.7. Statistical Analysis

The experiments were performed in triplicate and values were expressed as mean ± SD. One-way analysis of variance (ANOVA) was used when comparing emulsion droplet size, PDI and zeta potential value of SEOF. The differences between means were evaluated by Tukey’s test.

## 5. Conclusions

In conclusion, a SEOF was successfully prepared by using a lecithin-surfactant system. The use of lecithin in combination with surfactant blends helped develop a stable SEOF that can be dispersed in simulated GI fluid to form O/W emulsions with droplet sizes close to 200 nm. The GC-MS analysis demonstrated that oleic acid was the major fatty acid in SEOF which showed good fatty acid chemical stability. Moreover, the oil adsorption measurements indicated that a better aqueous dispersibility of SEOF could possibly assist increasing the contact area between oil droplets and the membrane surface. Although an enzymatic digestion of the self-emulsified oil may need to be further studied, improved adsorption of oil components on membrane could increase the contact time and potentially improve the biological uptake of essential fatty acids and oil soluble bioactives. In future studies, we will process SEOF into soft gelatin capsules and evaluate their physicochemical stability.

## Figures and Tables

**Figure 1:** Two different dietary oil/fat absorption mechanisms. The mechanism for conventional dietary oil absorption (upper pathway) consists of emulsification by pancreatic bile salts, digestion with lipase and translocation of fatty acid micelles to the intestinal epithelium. The mechanism for a proposed self-emulsified dietary oil absorption (lower pathway) consist of adsorption of nano-emulsion onto unstirred mucus glycocalyx layer, lipase digestion of the localized oil and the absorption of free fatty acids.

**Figure 2:** Ternary phase diagram showing the region of clear isotropic liquids (grey) for SEOF; normal scale (**a**) and close-up view of the isotropic region (**b**).

**Figure 3:** Appearance of tea seed oil (**left**) and SEOF (A1) (**right**).

**Figure 4:** GC-MS chromatograms of tea seed oil (**left**) and SEOF (A1) (**right**) after transesterification.

**Figure 5:** Appearance of membrane after performed in a Franz cell apparatus; tea seed oil (**top**) and SEOF (**down**).

**Figure 6:** SEM images of membrane surface after performed in Franz cell apparatus; blank (**a**) tea seed oil (**b**) and SEOF (**c**).

**Figure 7:** GC-MS chromatograms of oil extracted from membrane after performed with SEOF in the Franz cell apparatus.

**Table 1:** Emulsion droplet size, polydispersity index (PDI) and zeta potential (ZP) of SEOF.

Formula	Lecithin (%)	Surfactant Blends (%)	Droplet Size (nm) ^NS^	PDI	ZP (mV)
A1	3	0.1	216.34 ± 16.38	0.271 ± 0.058 ^ab^	−17.98 ± 1.63 ^a^
A2		2	208.20 ± 7.03	0.277 ± 0.048 ^b^	−7.78 ± 0.73 ^cd^
A3		4	220.42 ± 15.77	0.244 ± 0.029 ^ab^	−6.16 ± 0.63 ^d^
B1	6	0.1	225.29 ± 29.39	0.264 ± 0.022 ^ab^	−18.86 ± 2.57 ^a^
B2		2	209.30 ± 8.49	0.239 ± 0.022 ^ab^	−11.03 ± 1.77 ^bc^
B3		4	221.60 ± 20.00	0.195 ± 0.018 ^ab^	−7.85 ± 0.71 ^cd^
C1	9	0.1	222.74 ± 15.13	0.259 ± 0.022 ^ab^	−18.87 ± 1.45 ^a^
C2		2	212.42 ± 8.34	0.204 ± 0.031 ^ab^	−11.97 ± 1.30 ^bc^
C3		4	214.84 ± 9.15	0.190 ± 0.020 ^ab^	−8.99 ± 0.73 ^bcd^
D1	12	0.1	224.91 ± 23.79	0.239 ± 0.031 ^ab^	−20.39 ± 2.57 ^a^
D2		2	206.40 ± 3.00	0.175 ± 0.040 ^a^	−13.08 ± 1.44 ^b^
D3		4	208.51 ± 10.27	0.197 ± 0.010 ^ab^	−10.39 ± 1.35 ^bc^

All data are presented as mean ± SD (*n* = 3). NS = Not statistically different. Means in the same column followed by different letters (a–d) were significantly different (*p* < 0.05).

**Table 2:** Levels (%) of fatty acid composition obtained from tea seed oil and SEOF.

Sample	Palmitic Acid (C16:0)	Stearic Acid (C18:0)	Oleic Acid (C18:1)	Linoleic Acid (C18:2)
Tea seed oil	8.83 ± 0.13	1.37 ± 0.05	82.17 ± 0.10	7.64 ± 0.13
SEOF	9.01 ± 0.04	1.52 ± 0.07	80.64 ± 0.32	8.83 ± 0.29

All data are presented as mean ± SD (*n* = 3).

**Table 3:** The amount (g/100 g sample) of each fatty acid obtained from SEOF over the times (0, 1, 2, 3 months) at 30 °C.

Time (Month)	Fatty Acid Content (g/100 g of SEOF)			
	Palmitic Acid (C16:0)	Stearic Acid (C18:0)	Oleic Acid (C18:1)	Linoleic Acid (C18:2)
0	8.41 ± 0.03	1.63 ± 0.01	61.58 ± 0.46	11.34 ± 0.15
1	9.63 ± 0.09	1.80 ± 0.04	61.52 ± 0.35	11.50 ± 0.05
2	9.26 ± 0.07	1.91 ± 0.04	61.05 ± 0.55	11.66 ± 0.10
3	9.76 ± 0.05	1.81 ± 0.06	61.75 ± 0.54	11.57 ± 0.22

All data are presented as mean ± SD (*n* = 3).

## References

[1] Kumar A., Sharma S., Kamble R. (2010). Self emulsifying drug delivery system (SEDDS): Future aspects. Int. J. Pharm. Pharm. Sci..

[2] Shrivastava S., Yadav S.K., Verma S. (2014). Applications of self emulsifying drug delivery systems in novel drug delivery- a review. Afr. J. Basic Appl. Sci..

[3] Chu J., Cheng Y.L., Rao A.V., Nouraei M., Zarate-Muñoz S., Acosta E.J. (2014). Lecithin-linker formulations for self-emulsifying delivery of nutraceuticals. Int. J. Pharm..

[4] He L., Guo-ying Z., Huai-yun Z., Jun-ang L. (2011). Research progress on the health function of tea oil. J. Med. Plants Res..

[5] Su M.H., Shih M.C., Lin K.H. (2014). Chemical composition of seed oils in native Taiwanese Camellia species. Food Chem..

[6] Lv G.P., Aoli M., Zhou B., Zhao J. (2013). Development of a rapid and simple non-derivatization method to determine constituents and antioxidative capacity of camellia oils by HPTLC. Food Nutr. Sci..

[7] Kalepu S., Manthina M., Padavala V. (2013). Oral lipid-based drug delivery systems—An overview. Acta Pharm. Sin. B.

[8] O’Driscoll C.M. (2002). Lipid-based formulations for intestinal lymphatic delivery. Eur. J. Pharm. Sci..

[9] Mahapatra A.K., Murthy P.N., Swadeep B., Swain R.P. (2014). Self-emulsifying drug delivery systems (SEDDS): An update from formulation development to therapeutic strategies. Int. J. PharmTech Res..

[10] Gershanik T., Benita S. (2000). Self-dispersing lipid formulations for improving oral absorption of lipophilic drugs. Eur. J. Pharm. Biopharm..

[11] Eid A.M.M., Baie S.H., Arafat O.M. (2012). The effect of surfactant blends on the production of a novel *Swietenia macrophylla* oil self-nanoemulsifying system. Int. J. Pharm. Pharm. Sci..

[12] Athas J.C., Jun K., McCafferty C., Owoseni O., John V.T., Raghavan S.R. (2014). An effective dispersant for oil spills based on food-grade amphiphiles. Langmuir.

[13] Yuan J.S., Ansari M., Samaan M., Acosta E.J. (2008). Linker-based lecithin microemulsions for transdermal delivery of lidocaine. Int. J. Pharm..

[14] Acosta E.J., Nguyen T., Witthayapanyanon A., Harwell J.H., Sabatini D.A. (2005). Linker-based bio- compatible microemulsions. Environ. Sci. Technol..

[15] Al-Sabagh A.M., Emara M.M., El-Din M.R.N., Aly W.R. (2011). Formation of water-in-diesel oil nano-emulsions using high energy method and studying some of their surface active properties. Egypt. J. Petrol..

[16] Patel R.B., Patel M.R., Bhatt K.K., Patel B.G. (2013). Formulation consideration and characterization of microemulsion drug delivery system for transnasal administration of carbamazepine. Bull. Fac. Pharm. Cairo Univ..

[17] Avachat A.M., Patel V.G. (2015). Self nanoemulsifying drug delivery system of stabilized ellagic acid–phospholipid complex with improved dissolution and permeability. Saudi Pharm. J..

[18] Kohli K., Chopra S., Dhar D., Arora S., Khar R.K. (2010). Self-emulsifying drug delivery systems: An approach to enhance oral bioavailability. Drug Discov. Today.

[19] Zanchetta B., Chaud M.V., Santana M.H.A. (2015). Self-emulsifying drug delivery systems (SEDDS) in pharmaceutical development. J. Adv. Chem. Eng..

[20] Jantratid E., Janssen N., Reppas C., Dressman J.B. (2008). Dissolution media simulating conditions in the proximal human gastrointestinal tract: An update. Pharm. Res..

[21] Cascone S., Lamberti G., Titomanlio G. (2014). Designing *in vitro* systems to simulate the *in vivo* permeability of drugs. Transl. Med. UniSa.

